The article "DNA methylation-associated inactivation of TGFβ-related genes DRM/Gremlin, RUNX3, and HPP1 in human cancers" was retracted in 2013. Reasons: manipulated images; misconduct by an author; duplicated images.

# DNA methylation-associated inactivation of TGF*β*-related genes *DRM/Gremlin*, *RUNX3*, and *HPP1* in human cancers

**DOI:** 10.1038/sj.bjc.6602837

**Published:** 2005-10-18

**Authors:** M Suzuki, H Shigematsu, D S Shames, N Sunaga, T Takahashi, N Shivapurkar, T Iizasa, E P Frenkel, J D Minna, T Fujisawa, A F Gazdar

**Affiliations:** 1 Hamon Center for Therapeutic Oncology Research, University of Texas Southwestern Medical Center, Bld NB, Room 8206, 6000 Harry Hines Blvd., Dallas, TX 75390, USA; 2 Department of Thoracic Surgery, Graduate School of Medicine, Chiba University, 1-8-1 Inohana, Chuo-ku, Chiba 260-8670, Japan

**Keywords:** *DRM/Gremlin* (*CKTSF1B1*), *HPP1*, *RUNX3*, TGF*β*, methylation

## Abstract

The transforming growth factor *β* (TGF*β*)-signalling pathway is deregulated in many cancers. We examined the role of gene silencing via aberrant methylation of *DRM/Gremlin* and *HPP1*, which inhibit TGF*β* signalling, and *RUNX3*, which facilitates TGF*β*-signalling, of all genes that are thought to be tumour suppressors, are aberrantly expressed, and are thus thought to have important role in human cancers. We examined *DRM/Gremlin* mRNA expression in 44 cell lines and the promoter methylation status of *DRM/Gremlin*, *HPP1*, and *RUNX3* in 44 cell lines and 511 primary tumours. The loss of *DRM/Gremlin* mRNA expression in human cancer cell lines is associated with DNA methylation, and treatment with the methylation inhibitor-reactivated mRNA expression (*n*=13). Methylation percentages of the three genes ranged from 0–83% in adult tumours and 0–50% in paediatric tumours. Methylation of *DRM/Gremlin* was more frequent in lung tumours in smokers, and methylation of all three genes was inversely correlated with prognosis in patients with bladder or prostate cancer. Our results provide strong evidence that these TGF*β*-related genes are frequently deregulated through aberrant methylation in many human malignancies.

The transforming growth factor *β* (TGF*β*) superfamily of paracrine and autocrine signalling molecules regulates many intra- and extracellular functions, including development, proliferation, differentiation, extracellular matrix and bone formation, angiogenesis, and immune responses (Balemans and Van Hul, 2002; Gumienny and Padgett, 2002). The TGF*β* family includes TGF*β*s, bone morphogenetic proteins (BMPs), activins, and several other subfamilies. Transforming growth factor *β* family members and their receptors are expressed by many types of normal and malignant cells. Both upregulation and downregulation of TGF*β* family member signalling may occur in cancer cells during different stages of pathogenesis (de Caestecker *et al*, 2000; Teicher, 2001; Roberts and Wakefield, 2003). Downregulation frequently occurs early in tumour development and is associated with increased epithelial growth and inhibition of apoptosis, while upregulation is more frequent during later stages and is associated with increased angiogenesis, stromal remodelling, suppression of immune responses, and metastatic spread. These cellular changes may occur via deregulation of interaction with Smad proteins at the nuclear level, via increased secretion of ligands by tumour cells, and/or by inactivation of ligands by soluble or intracellular inhibitors (de Caestecker *et al*, 2000; Teicher, 2001; Roberts and Wakefield, 2003).

The article "DNA methylation-associated inactivation of TGFβ-related genes DRM/Gremlin, RUNX3, and HPP1 in human cancers" was retracted in 2013. Reasons: manipulated images; misconduct by an author; duplicated images.

A large number of soluble inhibitors of TGF*β* family members have been identified (Gumienny and Padgett, 2002). The *DRM/Gremlin* (*CKTSF1B1*) gene, a member of the Cerberus/Dan family of BMP-soluble antagonists (Pearce *et al*, 1999), was independently isolated by two groups (Topol *et al*, 1997; Hsu *et al*, 1998). Topol *et al* (1997) isolated *Drm* from a rat model in which they demonstrated that transfection of *Drm* induced apoptosis and inhibited growth in rat fibroblasts. Hsu *et al* (1998) isolated *Gremlin* in *Xenopus* and demonstrated that it was a secreted protein that functioned as a BMP antagonist. *DRM/Gremlin* has been reported to influence BMP2-associated signalling pathways stimulated by fibroblast growth factor (Zuniga *et al*, 1999) and platelet-derived growth factor (PDGF) (Ghosh Choudhury *et al*, 1999), and it also negatively modulates embryonic lung morphogenesis (Shi *et al*, 2001).

Although the importance of *DRM/Gremlin* has been demonstrated during development and in the pathogenesis of nephropathy (Zuniga *et al*, 1999; McMahon *et al*, 2000; Khokha *et al*, 2003), its role in cancer pathogenesis is poorly understood. Topol *et al* (2000) recently mapped the human homologue of *DRM/Gremlin* to chromosome 15q13–15 and demonstrated that *DRM/Gremlin* mRNA expression is downregulated in several human tumour types. These researchers also found that the *DRM/Gremlin* transcript is normally expressed only in healthy breast epithelium. While these findings suggest that *DRM/Gremlin* is a tumour suppressor gene (TSG), how it is silenced in cancer cells is not known.

The *HPP1* (TMEFF2) gene belongs to another, possibly unique, class of TGF*β* antagonists. *HPP1* is a transmembrane receptor containing two follistatin modules and a single epidermal growth factor (EGF)-like domain (Uchida *et al*, 1999). Follistatin, a secreted soluble inhibitor, binds and neutralises the activity of many TGF*β* family members, including BMPs and activins, as well as PDGF and vascular endothelial growth factor (Patel, 1998; Lin *et al*, 2003). The EGF-like domain in *HPP1* appears to be a ligand for c-erbB-4 (Uchida *et al*, 1999). Recently, Gery *et al* (2002) demonstrated that *HPP1* exhibits antiproliferative effects in prostate cancer cell lines . These researchers also demonstrated an inverse correlation between *HPP1* activity in prostate cancer xenografts and c-*Myc* expression (Gery and Koeffler, 2003). Two soluble forms of HPP1 protein that differ in the presence/absence of the EGF-like domain arise by proteolytic cleavage (Uchida *et al*, 1999). Currently, it is not known which isoforms of *HPP1* are responsible for its tumour suppressor function. *HPP1* maps to chromosome 2q32.3, where loss of heterozygosity (LOH) frequently occurs in a number of tumours types, including lung cancer and breast cancer (Otsuka *et al*, 1996; Huiping *et al*, 1999).

The article "DNA methylation-associated inactivation of TGFβ-related genes DRM/Gremlin, RUNX3, and HPP1 in human cancers" was retracted in 2013. Reasons: manipulated images; misconduct by an author; duplicated images.

*RUNX3* is a Runt domain transcription factor that interacts with Smad proteins, suggesting that it may play an important role in TGF*β* signalling. This gene is a candidate TSG localised to 1p36, a region commonly deleted in a wide variety of human cancers, including lung cancer and breast cancer (Ragnarsson *et al*, 1999; Girard *et al*, 2000).

DNA methylation in the 5′ region is emerging as the primary mechanism of TSG inactivation (Jones and Baylin, 2002; Suzuki *et al*, 2004). Aberrant methylation of the *HPP1* and *RUNX3* genes has been demonstrated in gastrointestinal and other human tumours (Liang *et al*, 2000; Young *et al*, 2001; Guo *et al*, 2002; Li *et al*, 2002; Sato *et al*, 2002; Shibata *et al*, 2002; Kato *et al*, 2003; Xiao and Liu, 2004).

Using a microarray strategy, we recently identified *DRM/Gremlin* as a gene that was differentially expressed in a non-small-cell lung carcinoma (NSCLC) cell line after treatment with a demethylating agent (5-aza-2′-deoxycytidine (5-Aza-CdR)). Interestingly, lung cancer cell lines frequently demonstrate LOH at this gene location (Girard *et al*, 2000).

In this study, we examined mRNA expression and methylation status of *DRM/Gremlin* in lung cancer, breast cancer, and malignant mesothelioma (MM) cell lines, as well as the methylation status of *DRM/Gremlin*, *HPP1*, and *RUNX3* in several primary malignant tumours.

## MATERIALS AND METHODS

### Cell lines and tumour samples

In all, 28 lung cancer cell lines (15 NSCLC cell lines and 13 small-cell lung cancer (SCLC)] cell lines), 10 breast cancer cell lines, and six MM cell lines that were established by our group (Phelps *et al*, 1996; Gazdar *et al*, 1998) and deposited in the American Type Culture Collection (Manassas, VA, USA), were used in this study. Cell cultures were grown in RPMI-1640 medium (Life Technologies Inc., Rockville, MD, USA) supplemented with 5% fetal bovine serum and incubated in 5% CO_2_ at 37°C. Cell lines established at the National Cancer Institute have the prefix NCI while those established at UT Southwestern Medical Center have the prefix HCC. Normal bronchial epithelial cells (NHBEC), normal mammary epithelial cells (NHMEC), and normal mesothelial cells (NMC) were cultured as reported previously (Suzuki *et al*, 2005), and normal trachea RNA was obtained from Clontech (Palo Alto, CA, USA).

The article "DNA methylation-associated inactivation of TGFβ-related genes DRM/Gremlin, RUNX3, and HPP1 in human cancers" was retracted in 2013. Reasons: manipulated images; misconduct by an author; duplicated images.

In all, 13 tumour cell lines with *DRM/Gremlin* methylation and lack of *DRM/Gremlin* gene expression were incubated in culture medium with 4 *μ*M (5-Aza-CdR) for 6 days, with medium changes on days 1, 3, and 5. Cells were harvested and RNA was extracted on day 6.

Primary lung tumours were obtained from the Chiba University Hospital, Japan, and other tumours were obtained from the hospital system of the University of Texas Southwestern Medical Center, after obtaining Institutional Review Board approval and signed informed consent. Samples were immediately frozen and stored at −80°C until use.

### Reverse transcriptase–PCR (RT–PCR) assay for *DRM/Gremlin*

An RT–PCR assay was used to examine *DRM/Gremlin* mRNA expression. Total RNA was extracted from samples with Trizol (Life Technologies, Rockville, MD, USA) following the manufacturer's instructions. The RT reaction was performed on 4 *μ*g total RNA with Deoxyribonuclease I and the SuperScript II First-Strand Synthesis using the oligo(dT) primer System (Life Technologies), and aliquots of the reaction mixture were used for subsequent PCR amplification. Primer sequences for *DRM/Gremlin* amplification were: forward, 5′-ACTCAGCGCCACGCGTCGAAA-3′; reverse, 5′-ACTGAGTCTGCTCTGAGTCATT-3′ (GenBank accession number AC090877; forward, nucleotides 52619–52639; reverse, nucleotides 65324–65345), and we confirmed that genomic DNA was not amplified with these primers which cross an intron. The amplification programme for the *DRM/Gremlin* transcript was 1 min at 94°C, 1 min at 60°C, and 1 min at 72°C for 40 cycles. The housekeeping gene *GAPDH* was used as an internal control to confirm the success of the RT reaction. Primer sequences for *GAPDH* amplification were: forward, 5′-CACTGGCGTCTTCACCACCATG-3′; reverse, 5′-GCTTCACCACCTTCTTGATGTCA-3′ (GenBank accession number NM_002046). These primer sequences were identical to the endogenous human target genes as confirmed by a BLAST search. PCR products were analysed on 2% agarose gels. Normal bronchial epithelial cells, NHMEC, NMC, and normal trachea were used as normal controls for RT–PCR.

### Map of the 5′ flanking region of *DRM/Gremlin* and bisulphite DNA sequencing

The locations of CpG dinucleotides, the MSP amplicon (region of MSP (RMSP)), and the area that underwent bisulphite DNA sequencing (region of bisulphite sequencing (RBSSQ)) in the 5′ region of *DRM/Gremlin* are shown in Figure 3. Bisulphite-treated DNA was PCR-amplified using the following primers: forward, 5′-TGTGATTTGTTGTGTATTTTAGG-3′; reverse, 5′-ATAATTCTTCACAATTCACCCC-3′ (GenBank accession number AC090877, 52248–52821, 574 bp). These primers were designed to exclude binding to any CpG dinucleotides to ensure amplification of both methylated and unmethylated sequences. PCR products were cloned into plasmid vectors using the Topo TA cloning kit (Invitrogen, Carlsbad, CA, USA) following the manufacturer's instructions. Five positive clones were purified from each test cell line using the Wizard Plus miniprep kit (Promega), and were then sequenced by the Applied Biosystems PRISM dye terminator cycle sequencing method (Perkin-Elmer Corp., Foster City, CA). This region included the MSP primer sites and amplicon and encompassed 77 CpG dinucleotides.

The article "DNA methylation-associated inactivation of TGFβ-related genes DRM/Gremlin, RUNX3, and HPP1 in human cancers" was retracted in 2013. Reasons: manipulated images; misconduct by an author; duplicated images.

### DNA extraction and methylation-specific PCR

Genomic DNA was obtained from cell lines, primary tumours, and normal cells by digestion with proteinase K (Life Technologies), followed by phenol/chloroform (1 : 1) extraction (Suzuki *et al*, 2003). DNA methylation patterns in the CpG island of *DRM/Gremlin* were determined by the methylation-specific PCR (MSP) method as reported as described previously (Herman *et al*, 1996). Primer sequences of *DRM/Gremlin* for methylated reaction were as follows: forward, 5′-ATTTAAACGGGAGACGGCGCG-3′; reverse, 5′-GACCAAAACCGCCGAAACTCG-3′; those for the unmethylated reaction were: forward, 5′-ATTTAAATGGGAGATGGTGTG-3′; reverse, 5′-AACCAAAACCACCAAAACTCA-3′. Primer sequences for amplification of *HPP1* and *RUNX3* for MSP have been previously described (Li *et al*, 2002; Sato *et al*, 2002). Briefly, 1 *μ*g genomic DNA was denatured by NaOH and modified by bisulphite. The modified DNA was purified using Wizard DNA purification kit (Promega), treated with NaOH to desulfonate, precipitated with ethanol and resuspended in water. PCR amplification was performed with bisulphite-treated DNA as a template using specific primer sequences for the methylated and unmethylated forms of the genes. DNA from peripheral blood lymphocytes (*n*=10) from healthy subjects (non-smoking) was used as negative controls for MSP assays. DNA from lymphocytes of a healthy volunteer treated with Sss1 methyltransferase (New England BioLabs, Beverly, MA) and then subjected to bisulphite treatment was used as a positive control for methylated alleles. Water blanks were included with each assay. Results were confirmed by repeating bisulphite treatment and MSP for all samples.

The article "DNA methylation-associated inactivation of TGFβ-related genes DRM/Gremlin, RUNX3, and HPP1 in human cancers" was retracted in 2013. Reasons: manipulated images; misconduct by an author; duplicated images.

### Data analysis

Statistical differences between groups were examined using Fisher's exact test, the chi-square test, and the Mann-Whitney test. Survival was calculated from the date of initial diagnosis until death or the date of the last follow-up (censored). Survival was analysed according to the Kaplan-Meier method, and differences in distribution were evaluated by means of the log-rank test. A *P*-value of less than 0.05 was defined as being statistically significant.

## RESULTS

### *DRM/Gremlin* mRNA expression in normal and malignant breast, lung, and mesothelial cells

We used RT–PCR to examine the expression of *DRM/Gremlin* (Table 1); representative examples are shown in Figure 1A. *DRM/Gremlin* mRNA was detected in NHBEC, normal trachea, NHMEC, and NMC, indicating that this gene is normally expressed in respiratory cells, breast epithelial cells, and mesothelial cells. However, loss of *DRM/Gremlin* expression was observed in 12/15 (80%) of NSCLC cell lines, 5/13 (38%) of SCLC cell lines, 5/10 (50%) of breast cancer cell lines, and 4/6 (67%) of MM cell lines (Table 1 and Figure 2).

### Bisulphite genomic DNA sequencing of the 5′ region of *DRM/Gremlin*

We sequenced bisulphite-treated DNA in the 5′ region of *DRM/Gremlin* to clarify any correlation between DNA methylation and gene silencing in various cancer cell lines. Using methylation-independent primers, we amplified and sequenced the 5′ region and exon 1 of the *DRM/Gremlin* gene (Figure 3). The 574-bp amplicon contains 77 CpG dinucleotides as well as exon 1. The translation start site is in exon 2. The G+C percentage is 74%, with a CpG ratio of 1. This region therefore satisfied the criteria for a CpG island (Gardiner-Garden and Frommer, 1987). Eight cell lines showed an excellent concordance between MSP and RT–PCR assay results and clonal sequencing results. Two normal tissues (normal lung and peripheral blood lymphocytes) also showed concordance between MSP assay and sequencing results. We developed MSP primers based on these sequencing results.

### DNA methylation of *DRM/Gremlin* in cell lines and tissues

The DNA methylation status of *DRM/Gremlin* in cell lines as assessed by MSP assays are detailed in Table 1 and Figure 3, and representative examples are illustrated in Figure 4. Methylation of *DRM/Gremlin* was absent in DNA from peripheral blood lymphocytes from healthy volunteers and in respiratory cells, breast epithelial cells, and mesothelial cells. In contrast, *DRM/Gremlin* methylation was detected in 11/15 (73%) of NSCLC cell lines, 4/13 (31%) of SCLC cell lines, 5/10 (50%) of breast cancer cell lines, and 4/6 (67%) of MM cell lines. Either the methylated or the unmethylated forms of the gene were present in most cell lines (37/44 (84%)), while both forms were present in the remaining seven (16%) cell lines. Overall concordance between *DRM/Gremlin* expression and methylation was 42/44 (95%).

The article "DNA methylation-associated inactivation of TGFβ-related genes DRM/Gremlin, RUNX3, and HPP1 in human cancers" was retracted in 2013. Reasons: manipulated images; misconduct by an author; duplicated images.

### Restoration of *DRM/Gremlin* expression in 5-Aza-CdR-treated cancer cells

A total of 13 tumour cell lines (five NSCLC, one SCLC, three breast cancer, and four MM) that showed loss of expression and methylation of *DRM/Gremlin* were cultured with 5-Aza-CdR. *DRM/Gremlin* expression was restored after treatment in all 13 cell lines (Figure 1B).

### DNA methylation of *DRM/Gremlin, HPP1*, and *RUNX3* in primary tumours and tissues and its correlation to clinicopathologic features

*DRM/Gremlin* is aberrantly methylated and downregulated in thoracic cancer cell lines. *HPP1* and *RUNX3* have also been shown to be aberrantly methylated in certain cancer types. These three genes are TGF*β* related and are all thought to be tumour suppressors. We next examined the methylation status of these three genes in primary tumours and tissues by MSP assay (Tables 2 and 3, Figure 4). Methylation of *DRM/Gremlin* was observed in 50% of lung cancer tissues (*n*=140), 54% of breast cancer tissues (*n*=37), and 60% of MM tissues (*n*=63), while methylation of *HPP1* in these tissues occurred at a frequency of 28, 35, and 35%, respectively, and methylation of *RUNX3* occurred at a frequency of 18, 22, and 33%, respectively. The methylation frequency for all three genes was significantly higher in adult tumours compared to paediatric tumours (*DRM/Gremlin*, *P*<0.0001; *HPP1*, *P*<0.0001; *RUNX3*, *P*<0.0001). Methylation of all three genes appeared to be tumour specific in all adult tumours, when compared to corresponding adjacent normal tissues (*P*<0.0001). Methylation of these genes was not detected in bronchial carcinoids.

In lung cancer tissue, *DRM/Gremlin* methylation was not associated with age, postsurgical stage, or prognosis, but it was associated with gender (male, 68/88 (77%); female, 18/35 (51%); *P*=0.008) and smoking history (smoker, 74/97 (76%); nonsmoker, 12/26 (46%); *P*=0.007). In breast cancer samples, methylation of *DRM/Gremlin* gene was associated with older age (*P*=0.009). In addition, the frequency of methylation for *RUNX3* was higher in estrogen receptor (ER)-positive cases than in ER-negative cases (ER positive, 8/22 (36%); ER negative, 0/8 (0%); *P*=0.02). In bladder cancer tissues, methylation of *DRM/Gremlin* was associated with poorer prognosis (*P*=0.026, log-rank test) (Figure 5). The frequencies of methylation for *DRM/Gremlin* and *HPP1* were higher in advanced-stage bladder cancer cases (stages III–IV) than in early-stage cases (stages 0–II, *P*=0.03 and 0.003, respectively). The frequency of methylation for *RUNX3* was higher in the presence of muscle invasion cases (20/39 (51%)) than in the absence of muscle invasion cases (4/18 (22%); *P*=0.048). In prostate cancer tissues, methylation of these three genes did not appear to be correlated with age, stage, Gleason score, or serum prostate-specific antigen level. However, *RUNX3* and *HPP1* methylation-positive status were associated with poorer disease-free prognosis (*P*=0.007 and 0.014, respectively; log-rank test).

The article "DNA methylation-associated inactivation of TGFβ-related genes DRM/Gremlin, RUNX3, and HPP1 in human cancers" was retracted in 2013. Reasons: manipulated images; misconduct by an author; duplicated images.

## DISCUSSION

*DRM/Gremlin* encodes a 184-amino-acid protein that is a member of the cysteine knot superfamily (Hsu *et al*, 1998). This protein has been highly conserved during evolution and it belongs to a novel family of BMP antagonists that includes the tumour suppressor DAN. The BMPs play a major role in bone formation and may facilitate bone metastases derived from prostate tumours (Masuda *et al*, 2003) as well as other cancers. DRM/Gremlin protein blocks the activity of BMP2, BMP4, and BMP7 with high affinity (Hsu *et al*, 1998; Merino *et al*, 1999) and possibly that of other growth factors in the TGF*β* superfamily. BMP2 is overexpressed in NSCLC tissues and has been shown to stimulate growth of A549 lung cancer cells (Langenfeld *et al*, 2003). DRM/Gremlin is also known to affect lung development (Shi *et al*, 2001). BMP2 exposure has been shown to increase phosphatase and tensin homolog (PTEN) protein levels in the breast cancer cell line MCF-7 (Waite and Eng, 2003). Blocking BMP signalling by overexpression of a dominant-negative type II BMP receptor inhibits the growth of human breast cancer cells (Pouliot *et al*, 2003). Recently, Chen *et al* demonstrated that overexpression of *Drm* in the tumour-derived cell lines Daoy (primitive neuroectodermal, HTB186) and Saos-2 (osteoblastic, HTB-85) transcriptionally activates *p21*^Cip1^ via a novel mechanism, independent of *p53* and both p38 and p42/44 MAP kinases, and inhibits neoplastic transformation (Chen *et al*, 2002). Thus, silencing of the *DRM/Gremlin* gene by DNA methylation may play a role in carcinogenesis both by affecting the cell cycle as well as by upregulation of BMP signalling.

We observed frequent methylation of *DRM/Gremlin* in many human adult cancer tissues and cell lines, and methylation appeared to be correlated with reduced *DRM/Gremlin* mRNA expression, suggesting that epigenetic phenomena (i.e., methylation and the related mechanism of histone deacetylation) were the major causes of gene silencing. Expression of these genes was reactivated following treatment with the demethylating agent 5-Aza-CdR, providing further evidence that methylation is indeed the silencing mechanism involved.

The article "DNA methylation-associated inactivation of TGFβ-related genes DRM/Gremlin, RUNX3, and HPP1 in human cancers" was retracted in 2013. Reasons: manipulated images; misconduct by an author; duplicated images.

Methylation of *DRM/Gremlin*, *HPP1*, and *RUNX3* appeared to be tumour specific in these cancer types when compared to corresponding adjacent normal tissues. Methylation of these genes in paediatric tumours was relatively rare, which is consistent with our previous reports (Harada *et al*, 2002). Methylation of these genes was not detected in bronchial carcinoids, which are lung tumours with relatively low invasive and metastatic potential. In a previous study, we found that the methylation profile of carcinoids was similar to that of SCLC, although the methylation frequencies of most genes were lower in carcinoids (Toyooka *et al*, 2001).

In our previous studies, we observed that the methylation frequencies of MGMT and GSTP1 in lung cancers were significantly higher in US and Australian cases than in those from Japan and Taiwan (Toyooka *et al*, 2003). In addition, methylation frequencies were either similar, or slightly higher (seldom significantly) in lung tumour cell lines than in primary tumours (Toyooka *et al*, 2001). In our present series, the primary lung tumours were from Japan while all of the other primary tumours as well as the cell lines were from the US. Although the methylation frequencies of *DRM/Gremlin* between primary tumours and cell lines for lung cancer, breast cancer, and MM were similar, further interethnic studies need to be performed to clarify this matter.

Although only a small number of breast cancer tissues were examined, tissues from older women showed a higher frequency of *DRM/Gremlin* methylation than did those from young women. Age-related methylation of TSGs has also been reported in colonic epithelium and cancer (Waki *et al*, 2003). Methylation of *DRM/Gremlin* was significantly more frequent in lung cancers arising in smokers compared to nonsmokers. We and others have noted a relationship between the methylation of certain genes, including *p16* and *APC*, as well as an increased overall methylation status in smoking-related lung cancers (Kim *et al*, 2001; Toyooka *et al*, 2003). In bladder cancers, *DRM/Gremlin* methylation-positive status was associated with poorer prognosis, while *RUNX3* and *HPP1* methylation-positive status was associated with poorer disease-free prognosis in prostate cancers. Although the number of samples tested in this study is too small to draw definitive conclusions, deregulation of TGF*β* signalling through hypermethylation of these genes may affect tumour progression as well as patients’ prognosis, resulting in more aggressive local and distant metastatic spread, including the bone. Of interest, bone metastases are frequent in the cancers examined in this study, particularly in SCLC, breast cancer, and prostate cancer.

The article "DNA methylation-associated inactivation of TGFβ-related genes DRM/Gremlin, RUNX3, and HPP1 in human cancers" was retracted in 2013. Reasons: manipulated images; misconduct by an author; duplicated images.

In conclusion, we found that two inhibitors and one modulator of TGF*β* signalling, *DRM/Gremlin*, *HPP1*, and *RUNX3*, respectively, are often methylated and thereby silenced in human cancers. Correlation between methylation of any of these genes with various clinicopathological features, including smoking status and survival, indicates that our findings may be of both biological and clinical relevance.

## Figures and Tables

**Figure 1:** RT–PCR for *DRM/Gremlin (CKTSF1B1)* expression in lung and breast cancer cell lines. (**A**) Representative examples of RT–PCR results for *DRM/Gremlin* expression. (**B**) Effect of 5-Aza-CdR treatment on *DRM/Gremlin*-negative cell lines with *DRM/Gremlin* methylation. Treatment with 5-Aza-CdR restored expression of *DRM/Gremlin* in all 13 methylated cell lines tested. Expression of the housekeeping gene *GAPDH* was measured as a control for RNA integrity. M, molecular size marker; LC, lung cancer; BC, breast cancer; MM, malignant mesothelioma; NEG, negative control (genomic DNA). Before (**B**) and after (**A**) treatment with 5-Aza-CdR.

**Figure 2:** *DRM/Gremlin (CKTSF1B1)* expression and methylation in tumour cell lines. Closed box, positive (POS) band detected; open box, negative (NEG) band detected; N, NSCLC cell line; S, SCLC cell line; B, breast cancer cell line; M, MM cell line; ND, not done.

**Figure 3:** The location and methylation status of methylated CpG dinucleotides in the region of *DRM/Gremlin* that underwent bisulphite genomic DNA sequencing (RBSSQ). Positive numbers indicate the nucleotide position from the transcription start site (TSS; indicated with an arrow). Thin vertical lines and the numbers indicate the positions of CpG dinucleotides in the RBSSQ. The horizontal closed bars between numbers indicate the positions of CpG dinucleotides included in the MSP primers. Open circles indicate unmethylated CpG sites and filled circles indicate methylated CpG sites.

**Figure 4:** Representative examples of MSP results for *DRM/Gremlin* in cell lines and primary tumours. (**A**) Representative examples of MSP results for *DRM/Gremlin* in lung cancer cell lines, breast cancer cell lines, and MM cell lines. *DRM/Gremlin* M, *DRM/Gremlin*-methylated form; *DRM/Gremlin* U, *DRM/Gremlin*-unmethylated; POS, positive control, that is, artificially methylated DNA; NEG, negative control (water blank). (**B**) Lung cancer (T), matched normal lung tissue (N), breast cancer (T), matched normal breast tissue (N). (**C**) MM, malignant pleural mesothelioma; BC, bladder cancer; PCa, prostate cancer; ML, malignant lymphoma. A visible band indicates amplification of a methylated form of a gene. Owing to contamination by normal tissues, either the unmethylated band only or both the methylated and unmethylated bands were present in several samples.

The article "DNA methylation-associated inactivation of TGFβ-related genes DRM/Gremlin, RUNX3, and HPP1 in human cancers" was retracted in 2013. Reasons: manipulated images; misconduct by an author; duplicated images.

**Figure 5:** Survival curves of bladder and prostate cancer cases. Survival was analysed according to the Kaplan–Meier method, and differences in distribution were evaluated using the log-rank test. (**A**) Overall survival curve according to *DRM/Gremlin* methylation status in bladder cancer cases (*n*=57). (**B**) Disease-free survival curve of prostate cancer cases (*n*=28) according to *RUNX3* and *HPP1* methylation status. Poorer overall and disease-free survival were observed in bladder cancer cases with *DRM/Gremlin* methylation and in prostate cancer cases with *RUNX3* and *HPP1* methylation.

**Table 1:** Methylation and expression of *DRM/Gremlin* in cell lines

	***DRM/Gremlin***	
**Samples**	**Expression (%)**	**Methylation (%)**
*Lung cancer cell lines (n*=*28)*		
NSCLC (*n*=15)	3 (20)	11 (73)
SCLC (*n*=13)	8 (62)	4 (31)
		
Breast cancer cell lines (*n*=10)	5 (50)	5 (50)
MM cell lines (*n*=6)	2 (33)	4 (67)
NHBEC (*n*=1)	1 (100)	0 (0)
NHMEC (*n*=2)	2 (100)	0 (0)
NMC (*n*=3)	3 (100)	0 (0)

MM=malignant mesothelioma; NHBEC=normal human bronchial epithelial cells; NHMEC=normal human mammary epithelial cells; NMC=normal human mesothelial cells.

**Table 2:** Methylation of *DRM/Gremlin*, *HPP1*, and *RUNX3* in human cancers

		**No. methylated (%)**		
**Samples**	**Total no.**	***DRM/Gremlin***	***HPP1***	***RUNX3***
*Adult tumours*	367			
Primary NSCLC				
Adenocarcinoma	60	22 (37)	18 (30)	13 (22)
Squamous cell carcinoma	51	40 (78)	15 (29)	8 (16)
Large cell carcinoma	6	5 (83)	4 (67)	4 (67)
Primary SCLC	5	3 (60)	2 (40)	0
Bronchial carcinoid	18	0	0	0
Malignant mesothelioma	63	38 (60)	22 (35)	21 (33)
Breast cancer	37	20 (54)	13 (35)	8 (22)
Prostate cancer	50	10 (20)	19 (38)	5 (10)
Bladder cancer	57	29 (51)	20 35)	24 (42)
Lymphoma	20	10 (50)	6 (30)	1 (5)
				
*Paediatric tumours*	150			
Osteosarcoma	10	1 (10)	0	5 (50)
Wilm’s tumour	25	0	0	0
Neuroblastoma	27	0	0	0
Rhabdomyosarcoma	17	1 (6)	0	0
Medulloblastoma	12	0	0	0
Hepatoblastoma	22	0	0	0
Ewing sarcoma	7	0	0	0
Retinoblastoma	30	0	0	0
				
*Normal tissues*	138			
Lung tissues^a^ and NHBEC	51	1 (2)	0	0
Mesothelial cells	3	0	0	0
Breast tissues^a^	23	0	0	0
Protate tissues^a^	4	0	0	0
Bladder tissues^a^	5	0	0	0
Peripheral blood lymphocytes^b^	14	0	0	0

a Adjacent to resected tumours.

b From healthy volunteers.

The article "DNA methylation-associated inactivation of TGFβ-related genes DRM/Gremlin, RUNX3, and HPP1 in human cancers" was retracted in 2013. Reasons: manipulated images; misconduct by an author; duplicated images.

**Table 3:** Clinicopathologic correlation with the methylation of *DRM/Gremlin*, *HPP1* and *RUNX3* in adult solid tumours

**Clinicopathologic features**	***DRM/Gremlin* methylation (%)**	***P* a**	***HPP1* methylation (%)**	***P***	***RUNX3* methylation (%)**	***P***
*Lung cancers*						
*Gender*						
Male (*n*=88^b^)	68 (77)	0.008	25 (28)	0.3	18 (20)	0.9
Female (*n*=35)	18 (51)		14 (40)		7 (20)	
						
*Age* c						
⩽65 (*n*=60)	42 (70)	0.9	19 (32)	0.9	13 (22)	0.8
>65 (*n*=63)	44 (70)		20 (32)		12 (19)	
						
*Smoking history*						
Nonsmoker (*n*=26)	12 (46)	0.007	8 (31)	0.9	5 (19)	
Smoker (*n*=97)	74 (76)		31 (32)		20 (21)	0.9
						
*Histology*						
Adenocarcinoma (*n*=60)	38 (63)		18 (30)		13 (22)	
Squamous cell ca. (*n*=51)	40 (78)		15 (29)		8 (16)	
Large cell ca. (*n*=6)	5 (83)		4 (67)		4 (67)	
Small cell ca. (*n*=5)	3 (60)		2 (40)		0 (0)	
Carcinoid (*n*=18)	0 (0)		0 (0)		0 (0)	
						
*Postsurgical stage*						
Stages I and II (*n*=52)	42 (81)	0.03	19 (36)	0.3	8 (15)	0.3
Stages III and IV (*n*=71)	44 (62)		20 (28)		17 (24)	
						
*Breast cancers*						
*Age*						
⩽53 (*n*=17)	5 (29)	0.009	3 (18)	0.08	2 (12)	0.2
>53 (*n*=20)	15 (75)		10 (50)		6 (30)	
						
*Postsurgical stage*						
Stages I and IIA (*n*=21)	9 (43)	0.1	5 (24)	0.2	5 (24)	0.9
Stages IIB and IIIA (*n*=16)	11 (69)		8 (50)		3 (19)	
						
*Estrogen receptor status*						
Positive (*n*=22)	14 (64)	0.4	11 (50)	0.08	8 (36)	0.02
Negative (*n*=11)	6 (55)		2 (18)		0 (0)	
						
*Progesterone receptor status*						
Positive (*n*=20)	13 (65)	0.4	10 (50)	0.1	7 (35)	0.08
Negative (*n*=13)	7 (54)		3 (23)		1 (8)	
						
*Bladder cancers*						
*Gender*						
Male (*n*=36)	19 (53)	0.8	12 (33)	0.8	14 (39)	0.6
Female (*n*=21)	10 (48)		8 (38)		10 (48)	
						
*Age*						
⩽67 (*n*=29)	14 (48)	0.8	10 (34)	0.9	12 (41)	0.9
>67 (*n*=28)	15 (54)		10 (36)		12 (43)	
						
*Grade*						
Grades 1 and 2 (*n*=13)	5 (38)	0.5	2 (15)	0.2	2 (15)	0.05
Grade 3 (*n*=43)	23 (53)		17 (40)		21 (49)	
						
*Growth pattern*						
Nonpapillary (*n*=26)	15 (58)	0.4	10 (38)	0.8	13 (50)	0.3
Papillary (*n*=31)	14 (45)		10 (32)		11 (35)	
						
*Muscle invasion*						
Noninvasion (*n*=18)	7 (39)	0.3	3 (17)	0.07	4 (22)	0.048
Invasion (*n*=39)	22 (56)		17 (44)		20 (51)	
						
*Stage*						
Stages 0–II (*n*=16)	4 (25)	0.03	1 (6)	0.003	3 (19)	0.1
Stages III and IV (*n*=30)	18 (60)		15 (50)		14 (47)	
						
*Prostate cancers*						
*Age*						
⩽64 (*n*=27)	6 (22)	0.7	7 (26)	0.2	1 (4)	0.2
>64 (*n*=26)	4 (15)		12 (46)		4 (15)	
						
*Gleason score*						
⩽6 (*n*=22)	6 (27)	0.3	11 (50)	0.2	1 (5)	0.4
⩾7 (*n*=28)	4 (14)		8 (29)		4 (14)	
						
*Preoperative serum PSA* d						
⩽7.5 ng/ml (*n*=25)	5 (20)	0.7	8 (32)	0.9	2 (8)	0.9
⩾7.5 ng/ml (*n*=22)	3 (14)		7 (32)		2 (9)	

a Fisher’s exact probability test.

b Detailed data were available on the number in parentheses.

c Devided by median age.

d Prostate-specific antigen.
